RETRACTED

# Evaluation and Stratification for Chinese International Education Quality with Deep Learning Model

**DOI:** 10.1155/2022/9627116

**Published:** 2022-05-23

**Authors:** Min He

**Affiliations:** Department of Basic Education and Research, Shaanxi Police Vocational College, Xi'an 710021, China

## Abstract

In the process of human communication, language learning and communication play a fundamental, leading, broad, and long-lasting role. It serves as a link and a bridge between countries and peoples, allowing for greater understanding and camaraderie. The significance of Chinese in international commercial and cultural exchanges has been more obvious in the current era, as China's comprehensive strength continues to improve. Its cultural value and practical value have been continuously improved, the international community has an increasing demand for learning Chinese, and the cause of international Chinese language education has developed rapidly. China must strengthen the international dissemination of Chinese, so that the world can better understand and accept China, so that China can better integrate into the world. In this context, how to evaluate and stratify the quality of Chinese international education has become an important research topic. Relying on the hot deep learning technology in recent years, this work designs a neural network for evaluating the quality of international Chinese education. The content of this work is as follows: aiming at the serious defect of the current mainstream feature classification network that only uses the top-level features extracted by a single convolution layer to classify, which leads to the loss of classification accuracy. A multiscale feature pyramid fusion network is built in this paper, starting with the working mechanism of a convolutional neural network. It is capable of fully extracting and combining the representations of the network's shallow and deep outputs, based on first- and second-order characteristics of global and local discriminative region information. Second, the network structure has the bottleneck layer module and the batch normalization layer module, both of which are made up of varying numbers of 1 × 1 convolution kernels.

## 1. Introduction

Language learning and communication play a fundamental, leading, extensive, and lasting role in human communication and are bridges and bonds for deepening understanding and friendship between different countries and peoples. In the new era, with the continuous enhancement of China's comprehensive strength, the role of Chinese in international trade and cultural exchanges has become increasingly apparent. Its cultural value and practical value have been continuously improved, and the international community has an increasing demand for learning Chinese. Teaching Chinese to Speakers of Other Languages (TCSOL) is an emerging discipline that emerged in response to the rapid development of China's national strength to meet the needs of international communication of Chinese language. It was established in 2008. Teaching Chinese as a foreign language is based on coming in, while teaching Chinese as a foreign language is based on going out [1–5].

RETRACTED

In the past ten years, China's international Chinese language education has achieved amazing results. Teaching Chinese as a foreign language has gone further and further in the field of going global, and it is also closely aligned with many major national strategies. The main way for international Chinese language education to cooperate with the national strategy is to support countries around the world to cultivate local talents who are proficient in Chinese and understand Chinese culture, actively carry out Chinese cultural teaching and exchange activities, and help create a good environment for public diplomacy and cultural diplomacy. Through the subtle international education of Chinese and Chinese culture, it cultivates a large number of international friendly people who know and are friendly to China in a subtle and silent way and contributes to the promotion of China's international soft power. Therefore, the study of Chinese language education has become an indispensable research topic, which has very important theoretical and practical significance [6–10].

Teaching Chinese to Speakers of Other Languages is developing rapidly in both talent training and teaching research and is in a period of vigorous development. It can be seen that a scientific and systematic summary and analysis of the quality of education is a very important part of the field of Chinese language education research. Through the evaluation of education quality, stratified education can also be carried out. Dynamic stratified education teaches students according to their aptitude. It teaches on the premise of different personality characteristics. It can not only fully mobilize enthusiasm and initiative but also promote personality development, which has great advantages. At the same time, the dynamic layered teaching technique and the requirements of excellent education tend to be consistent; so, it is in line with the current teaching method reform and development. One of the foundations for the topic selection of this study [11–15] is the introduction of dynamic stratified teaching methods in teaching, organically merging with individual differences.

Neural network and deep learning is a very popular research method, and it has a solid theoretical foundation and powerful practical tools. Therefore, using deep learning as a means to analyze the quality of international Chinese language education is of great significance in detecting the hotspots and frontiers of the subject and choosing the direction of scientific research. On the one hand, it can make up for the inadequacy of the current deep learning analysis and research on Chinese international education in China. Through in-depth learning analysis, a new way of understanding Chinese international education research is formed. On the other hand, it can also summarize the achievements of the development and research of Chinese international education over the years, summarize the development law of the discipline, and provide information reference for Chinese experts and scholars in the research of the discipline theory. In this context, this work relies on the hot deep learning technology in recent years to design a neural network for evaluating the quality of Chinese international education. Its essence is a classification and identification network, and it is used for hierarchical research.

RETRACTED

The paper's organization paragraph is as follows: the related work is presented in Section 2.  Section 3 analyzes the design of application model.  Section 4 discusses the experiments and results. Finally, in Section 5, the research work is concluded.

## 2. Related Work

Reference [16] looked assessed the Chinese pronunciation of native English-speaking students from Europe and the United States, as well as their acquisition of Chinese phonetic changes. It also evaluates the influence of mother tongue, learning environment, and other aspects on its Chinese pronunciation based on its pronunciation. Reference [17] compares the initials, finals, and tones with the students' target language in the form of a survey report, finds out the reasons for the errors, and puts forward teaching suggestions. Reference [18] took foreign high school Chinese learners as the survey object and investigated the Chinese learning needs of these students. Reference [19] studies the needs of Chinese language learning at the Confucius Institute in Phuket, Thailand, and summarizes the completion of the work of the Confucius Institute. It includes the construction of Confucius Institutes/Classrooms, the construction of teaching staff, the compilation of local textbooks, the organization of international cultural activities, and the construction of online Confucius Institutes, as well as work plans and priorities. Literature [20] believes that the current scale of Confucius Institutes in China is developing steadily, the quality of running schools is constantly improving, the functions of running schools are constantly expanding, and the operating mechanism is gradually improving. At the same time, some suggestions and requirements are put forward for the future development of Confucius Institutes. Literature [21] emphasized the practical application value of Chinese language and the critical role of Confucius Institutes as incubators, predicting that Confucius Institutes' future development prospects would be broader. The literature [22] outlines the unique condition of studying in China, as well as the significant impact of the Belt and Road national policy on studying there. Literature [23] takes students whose immediate family members can speak Chinese in foreign schools as the research object, analyzes their different learning motivations, and puts forward different learning suggestions for different motivations. Reference [24] takes Confucius Institutes as the object of investigation and analyzes the current situation of Chinese language learning. It made a general exposition and analysis of the development status, existing problems, and future trends of Confucius Institutes based on the exchange materials of the 2nd Confucius Institute Conference, the relevant content of the Hanban website, and related articles. Literature [25] proposes that in the entire construction process of Confucius Institutes, innovative means must be used to continuously solve problems arising in the development and to continuously improve the effect of running schools. The Confucius Institute has become the brightest brand that reflects China's soft power. It is necessary to truly understand the soft power connotation of the Confucius Institute.

RETRACTED

According to Literature [26], focus should be devoted to the development of a comprehensive applied linguistics curriculum in the undergraduate course of Chinese international education. The viewpoints of undergraduate students majoring in Teaching Chinese to Speakers of Other Languages on the evolution of the major, future careers, and their comprehension of Chinese language teachers were explored in reference [27]. Literature [28] proposed a set of policies to encourage undergraduates studying in Chinese to work for Speakers of Other Languages. Taking the graduation thesis of the Master of Teaching Chinese to Speakers of Other Languages as the survey object, the subject selection of the thesis was poor in the examination. Literature [29] comprehensively investigates the current situation of Chinese talent courses in the majors of TESOL majors in four colleges and universities. Through the combination of questionnaire survey method, interview method, and other survey methods, this paper deeply analyzes the shortcomings and deficiencies in the curriculum setting of Chinese talent class. And trace back to the root of the problem and put forward reasonable suggestions for the improvement of Chinese talent courses from the aspects of colleges' attention, course offering, teachers' teaching, and students' learning. Literature [30] proposes that we should establish and enhance the subject awareness of teaching Chinese as a foreign language, strengthen the theoretical construction of teaching Chinese as a foreign language, and improve the quality of Chinese teaching that requires high-quality teachers, high-quality Chinese textbooks, and efficient teaching methods. Literature [31] proposed to strengthen the study of language acquisition laws and teaching methods to improve Chinese teaching. For the cultivation of the Master of Teaching Chinese to Speakers of Other Languages, not only skilled teaching skills are required but also good research quality. Literature [32] proposed that the principles of combining theory and practice and paying equal attention to knowledge transfer and skill training should be adopted in the process of master's degree training in Teaching Chinese to Speakers of Other Languages. We should emphasize the teaching of Chinese characters and knowledge of Chinese culture in specific courses, as well as the teaching of fundamental concepts and methods of foreign language teaching and the promotion of crosscultural teaching ability.

RETRACTED

## 3. Method

This chapter will deeply study and analyze the key factors that affect the classification performance of the existing mainstream classification evaluation models. Combined with the idea of multiscale feature pyramid, the classical algorithm is improved. Three high-performance and end-to-end Chinese international education quality evaluation models are constructed.

### 3.1. CNN

Compared with artificial neural network, convolutional neural network (CNN) simulates the biological mechanism of animal visual cortex. It adopts operations such as local connection, weight sharing, and downsampling, so that the network has certain invariance to the translation, distortion, and distortion of the image and easy to train and optimize. CNN is a multilayer feed-forward neural network, generally including input layer, convolution layer, pooling layer, fully connected layer, and output layer. The feature map of each layer is composed of a two-dimensional plane composed of multiple independent neurons. By setting multiple different convolution kernels to perform convolution operations, more new and different two-dimensional feature map information is extracted. After the convolution operation, through the activation function processing, the extracted feature information is pooled to retain the most significant features and enhance the robustness of the network. After multiple convolution and pooling operations, the extracted features are sent to the fully connected layer, and the mathematical statistics method is applied to construct a classifier to complete the classification and obtain the final output result.

RETRACTED

The role of the convolutional layer in the deep convolutional neural network is to extract new feature information from the input feature map and provide the next layer as input, which plays the role of layer advancement and feature extraction. The convolution kernel is a weight matrix. The setting of the parameters of the convolution kernel is very critical, involving the size, number, and step size of the convolution kernel. The settings of these parameters will affect the recognition accuracy of the model. The working principle of the convolution layer is to perform an inner product operation on the input feature map and the convolution kernel, and the convolution kernel performs a sliding window calculation on the input feature map. It maps the feature information in the kernel range into a new information and forms a new feature map as the input of the next layer. The size of the convolution kernel is the size of the receptive field sliding window. The larger the convolution kernel, the richer the extracted features, but at the same time, the number of parameters will increase sharply. The step size is the magnitude of the sliding window movement. The larger the step size, the smaller the size of the output feature map and the less information it contains. The smaller the step size, the more swipes, and the slower the network training. The convolution kernel can be regarded as a feature extractor, and different convolution kernels can extract different feature information in the input feature map. Therefore, the network can obtain a variety of different features at the same position in the image by increasing the number of convolution kernels, enrich the features learned by the model, and improve the cognitive ability of the model. The convolution operation is as follows:

(1) $$\begin{array}{c} x_{j}^{l}=f\left(\underset{j}{\sum }x_{i}^{l-1}*w_{ij}^{l-1}+b_{i}^{l}\right). \end{array}$$

After the convolution operation, the nonlinear output of the feature information is obtained through the activation function*f*, and the nonlinear transformation of the feature information is realized. This is a good way to solve classification problems that are tough to solve using linear classification [27]. The following are some of the most widely used activation functions:

(2) $$\begin{array}{c} \text{Sigmoid}\left(z\right)=\frac{1}{1+\exp\left(-z\right)},\\ \text{Tanh}\left(z\right)=\frac{\exp\left(z\right)-\exp\left(-z\right)}{\exp\left(z\right)+\exp\left(-z\right),}\\ \text{ReLU}\left(z\right)=\max\left(0,z\right). \end{array}$$

The pooling layer obtains the representative features in the local area image patch by downsampling. It further abstracts and reduces the dimension of the input feature map, reducing the computational cost. It can play the role of secondary feature extraction while reducing the dimension of the feature map. If the network does not change the size of the feature map during operation, it will increase the computational complexity of the convolutional layer and the parameter complexity of the fully connected layer. This will have a greater impact on the training of the network, making it difficult for the network to converge or even overfitting. The pooling layer can reduce the redundancy of features to a certain extent while reducing the size of the feature map. The pooling operation is similar to the convolution operation, using a pooling function without weight parameters. It begins in the upper left corner of the input feature map, slides to the right or down with a set step size, and outputs after pooling the pixels of the associated window block. The following is the calculating formula:

(3) $$\begin{array}{c} x_{j}^{l}=f\left(\beta \times \text{down}\left(x_{i}^{l-1}\right)+b_{j}^{l}\right). \end{array}$$

The most commonly used pooling methods are average pooling and max pooling. Average pooling is similar to the effect of the mean filter, which has a smoothing effect and can effectively avoid the influence of noise points, but it is easy to lose texture edge features. Since max pooling can reduce the mean deviation caused by the convolution operation, it can better adapt to texture features. The pooled features discard irrelevant details and only retain the main feature information that is effective for the task, which enables CNN to have a certain tolerance for changes in image translation, tilt, scale scaling, etc. The pooling layer only reduces the scale of a single feature map through the pooling kernel, retaining important feature details, and does not need to extract new features like the convolutional layer. Therefore, the number of feature maps remains unchanged after passing through the pooling layer.

RETRACTED

The function of the fully connected layer is to map the feature information obtained by operations such as convolution and pooling in front of the layer into the label space of the sample. Because the feature expression obtained by multiple convolutions and pooling of the convolutional neural network is still 3-dimensional, at this time, in order to calculate the gradient, the 3-dimensional feature expression must be corresponding to the 1-dimensional label. Therefore, a fully connected layer is required to convert 3-dimensional features into 1-dimensional space. The neurons in the fully connected layer are fully connected, and the output of all neurons in the previous layer will be used as the input of each neuron in this layer, but the neurons in the same layer are not connected to each other. The calculation method is as follows:

(4) $$\begin{array}{c} x_{j}^{l}=f\left(\underset{i}{\sum }x_{i}^{l-1}*w_{ij}^{l-1}+b_{i}^{l}\right). \end{array}$$

### 3.2. Multiscale Feature Pyramid Fusion Network

This section proposes an efficient multiscale feature pyramid fusion network (MSFPFN).  Figure 1 shows the MFPF network structure. The network framework can fully extract the first-order and second-order features of the global and local discriminative regional information that characterize the characteristics of international Chinese education for the final evaluation process, so as to effectively enhance and improve the performance of the basic network. At the same time, part of the network layer of the dual-channel VGG16-D network is used as the basic feature extractor to build the B-CNN model and the CBP model based on the low-dimensional approximation method of the Tensor Sketch kernel function as the basic network to build the network framework.

The network first uses the first 14 layers of two symmetric VGG16-D networks to build a two-way feature extractor. Afterwards, the feature maps output by the last two convolutional layers of the two-way feature extractor are used to extract different forms of second-order features across layers in the form of symmetry and intersection. At the same time, the feature maps output by the last three convolutional layers of the single-channel VGG16-D network are fused in the form of adding corresponding position elements to obtain first-order features. This first-order feature is then downsampled by the pooling layer, and the dimensionality reduction is performed by the mapping operation of the fully connected layer. Finally, the obtained first-order dimensionality reduction features that can represent the global information of the data and the second-order features with the characteristics of target discriminative region localization and identification are subjected to concat splicing and fusion operation and then sent to the Softmax classifier. At the same time, the MSFPFN network framework can also be extended to use other CNN networks with more advanced structure and better classification performance, such as ResNet and DenseNet, as the basic feature extractor to build. However, because the basic feature extractor chosen has a significant impact on the network model's final classification performance, it is necessary to avoid repeating related experiments and take into account the restricted computational resources. The goal of the related comparative experiments is to confirm that the proposed MSFPFN network framework's discriminative accuracy gain over the basic network comes from the first-order and second-order fusion features, which can effectively characterize the data's global and local discriminative region information, rather than merely using the improved classification performance of the underlying feature extractor. Therefore, in the research work of this paper, only part of the network layer of the VGG16-D network is used as the basic feature extractor to construct a high-performance Chinese international education quality assessment model. MSFPFN's specific parameters are listed in Table 1.

RETRACTED

### 3.3. Dimensionality Reduction Multiscale Feature Pyramid Fusion Network

As the dimension of the extracted bilinear features is higher, the computational complexity of the dimensionality reduction operation increases. And the more GPU memory resources are consumed during the network training process. Therefore, it is urgent to build a high-performance network framework based on feature dimensionality reduction. The Inception module has an excellent local topology network structure by using dense component connections instead of local sparse connections. Many design ideas used in the Inception module have had a profound impact on the construction of subsequent CNN models.

The Inception module adds several convolution and pooling bypass branches based on the convolutional sparse connection structure of the original direct connection. Feature maps representing different semantic information of the data are extracted by using parallel combination of convolution kernels of different sizes. Afterwards, these feature maps are subjected to concat splicing and fusion operation and then used as the input of subsequent network layers. In the Inception module, each bypass branch uses a 1 × 1 convolution kernel. It can effectively realize the combination of spatial feature information in the dimension direction of the input feature map channel and can perform data dimension reduction in a way of reducing the number of feature map channels. At the same time, the ReLU activation unit will be followed closely to add more nonlinear transformations to the network to improve the generalization ability of the model. In addition, the network layer constructed by the 1 × 1 convolution kernel is also called the bottleneck layer, which can be used to reduce the number of channels of the feature map first and then expand to the corresponding depth as needed.

RETRACTED

Based on the advantages of the bottleneck layer, this section embeds different numbers of bottleneck layer modules in the two-way feature extraction network of the MSFPFN network to construct a more efficient dimensionality reduction multiscale feature pyramid fusion network (MSFPFN-DR).  Figure 2 shows the network structure. The network structure of the two is similar, and the feature fusion method is the same. The main difference is that the MSFPFN-DR network, respectively, adds two different numbers of bottleneck layer modules after the last three convolutional layers of the two-way feature extractor VGG16-D network. It is used to reduce the dimension of the extracted first-order and second-order features to reduce the computational complexity of the network model. The subsequent first-order feature extraction operations and second-order feature extraction operations are similar to those of the MSFPFN network, with the exception that the dimensionality reduction mapping operation of the bottleneck layer module is added to the input part, demonstrating the MSFPFN-DR network framework's scalability even further.

### 3.4. DRMSFPFN with BN Layer

The great nonlinear fitting ability of the deep CNN model is complemented with a large number of parameters. When utilizing stochastic gradient descent for network model training, there are a few apparent hazards to be aware of. The initial learning rate, learning decay rate, each network layer's initialization weight, and the dropout usage ratio, for example, are all parameters that must be manually specified. These parameters have a significant impact on the network model's ultimate training performance. These vast quantities of parameter tweaking effort, on the other hand, are time and labor-intensive. In response to this problem, researchers have proposed an efficient BN layer module to solve this problem. The BN layer module can be used to accelerate the training convergence speed of the network, prevent overfitting, and effectively avoid the gradient disappearance or explosion problem during deep network training. The calculation of BN is as follows:

(5) $$\begin{array}{c} {x_{i}}^{\prime }=\frac{\left(x_{i}-\mu_{B}\right)}{\sqrt{\sigma^{2}+\varepsilon }},\\ y=\alpha {x_{i}}^{\prime }+\beta . \end{array}$$

At the same time, the BN layer module is usually added before the ReLU activation unit of each network layer when used in the CNN network. The feature maps extracted from each layer are first normalized and then nonlinearly mapped to smoothly accelerate the training convergence process of the network model.  Figure 3 shows the network structure changes before and after adding the BN layer module.

RETRACTED

Based on the benefits of the BN layer module, this part places the BN layer module before each MSFPFN-DR network layer ReLU activation unit to create the MSFPFN-DR-BN network, which improves the network's performance even more.

## 4. Experiment

### 4.1. Implementation Details

For experiments, this work uses a data collection that was created by the author. The data set contains a total of 87,314 samples, with 59,731 samples serving as the training set and 27,583 samples serving as the test set. Each sample's features are the appropriate evaluation indicators of Chinese international education quality, and the label is the quality level, which is then stratified according to the quality level. It should be emphasized that this work converts feature data into two-dimensional image data and views Chinese international education quality assessment as an image classification task. The experimental environment used in this work is shown in Table 2.

### 4.2. Training Convergence Evaluation

In deep learning, network training is a necessary and important process. The convergence of training directly affects the subsequent testing of the network. In order to evaluate the training process of the network, this work analyzes the losses in different stages of training. The experimental results are illustrated in Figure 4.

As the network training progresses, the loss gradually decreases. But when the epoch is 120, the loss value no longer decreases and tends to converge. This preliminarily shows the feasibility of the MSFPFN-DR-BN network designed in this paper.

### 4.3. Comparison of Different Methods

To further verify the effectiveness of MSFPFN-DR-BN, it is compared with other evaluation methods. The compared methods include RBF, SVM, and BP network, and the experimental results are illustrated in Table 3.

Compared with other methods in the table, MSFPFN-DR-BN can obtain 95.1% precision and 93.3% recall. It corresponds to the highest performance, which demonstrates the effectiveness and correctness of the method.

### 4.4. Multiscale Feature Fusion Evaluation

In this work, features of different scales are fused in order to extract more discriminative features. To verify the effectiveness of this strategy, this work conducts comparative experiments to compare the evaluation performance without feature fusion and when feature fusion is used. The experimental results are illustrated in Figure 5.

RETRACTED

Compared with single-scale features, using multiscale feature fusion can achieve 2.3% precision and 1.6% recall improvement. It can thus prove the effectiveness of this work using this feature fusion strategy.

### 4.5. Bottleneck Module Evaluation

This work adopts the bottleneck module to reduce the dimension of the network to speed up network training. In order to verify the effectiveness of this dimensionality reduction strategy, this work conducts comparative experiments to compare the evaluation performance without using the bottleneck module and using the bottleneck module, respectively. The experimental results are illustrated in Table 4.

It can be seen that after using the dimensionality reduction module, the training time of the network is greatly reduced, and the precision and recall are improved to varying degrees. This proves the correctness and feasibility of using this strategy in this work.

### 4.6. BN Module Evaluation

This work uses the BN module to optimize the network structure and extract more effective features. To verify the effectiveness of this strategy, the evaluation performance without and with BN is compared. The experimental results are illustrated in Figure 6.

Compared with not using the BN module, after using this strategy, the network can obtain 1.4% precision improvement and 1.2% recall improvement. This proves that the use of BN structure can effectively improve the evaluation performance.

## 5. Conclusion

After more than ten years of unrelenting work, Chinese foreign communication has reached its pinnacle. The international Chinese language education market is now in good shape and has a bright future ahead of it. The number of students has also increased, and cultural exchange programmers have become more varied and colorful. At the same time, the development of the Chinese domestic foreign education market is excellent. A growing number of colleges and institutions are offering undergraduate and master's degrees in Teaching Chinese to Speakers of Other Languages, and the number of international students in China is at an all-time high. Domestic and foreign Chinese language training institutions have already entered the initial stage, the market scale has continued to expand, and the brand concentration has gradually increased. The good development status of the Chinese international education market in China will lay a solid foundation for the international dissemination of Chinese in the future. In this context, how to evaluate and stratify the quality of Chinese international education has become an important research topic. This work designs a neural network for evaluating the quality of Chinese international education and conducts a hierarchical research based on this. Aiming at the common defects of existing mainstream network models, this paper improves the model by combining the idea of multiscale feature pyramid. To begin, we offer a network framework with high evaluation performance that can fully extract the first-order and second-order features of global and local discriminative area information to effectively enhance and improve the baseline model's classification performance. Second, due to the high dimension of the second-order features retrieved by the network and the computational cost, a bottleneck layer module made up of numerous 1 × 1 convolution kernels is integrated in the network structure to improve performance. In order to achieve effective dimensionality reduction of multilayer features, reduce the number of parameters of the model and improve the inference speed of the model. Finally, in order to effectively avoid and prevent the overfitting problem that is easy to occur in the deep network training process, BN layer modules are embedded before the ReLU activation units of each network layer to smoothly accelerate the training convergence process of the network model. Comprehensive and systematic experiments verify the effectiveness of this work.

RETRACTED

## Figures and Tables

**Figure 1:** The structure of MSFPFN.

**Figure 2:** The structure of MSFPFN-DR.

**Figure 3:** The network structure after adding the BN layer.

**Figure 4:** Training loss.

**Figure 5:** Multiscale feature fusion evaluation.

**Figure 6:** BN module evaluation.

**Table 1:** The detailed parameters of MSFPFN.

Layer	Kernel size	Kernel number	Input size
Conv1-1	3 × 3	64	448 × 448 × 3
Conv1-2	3 × 3	64	448 × 448 × 64
Maxpool1	2 × 2	—	448 × 448 × 64
Conv2-1	3 × 3	128	224 × 224 × 128
Conv2-2	3 × 3	128	224 × 224 × 128
Maxpool2	2 × 2	—	112 × 112 × 128
Conv3-1	3 × 3	256	112 × 112 × 128
Conv3-2	3 × 3	256	112 × 112 × 256
Conv3-3	3 × 3	256	112 × 112 × 256
Maxpool3	2 × 2	—	56 × 56 × 256
Conv4-1	3 × 3	512	56 × 56 × 256
Conv4-2	3 × 3	512	56 × 56 × 512
Conv4-3	3 × 3	512	56 × 56 × 512
Maxpool4	2 × 2	—	56 × 56 × 512
Conv5-1	3 × 3	512	28 × 28 × 512
Conv5-2	3 × 3	512	28 × 28 × 512
Conv5-3	3 × 3	512	28 × 28 × 512
Maxpool4	2 × 2	—	28 × 28 × 512
FC1	—	1	28 × 28 × 512
FC2	—	1	262244
Softmax	—	1	16484

**Table 2:** Experimental environment.

Item	Parameter
Operating system	Ubuntu 18.04
CPU	Intel(R) Xeon(R) CPU E5-2620 v4 @ 2.10GHz
Memory	32G
Graphics card	NVIDIA GeForce GTX 1080Ti
Framework	PyTorch

**Table 3:** Comparison of different methods.

Method	Precision	Recall
RBF	85.30	82.80
SVM	89.90	87.20
BP	92.70	91.60
MSFPFN-DR-BN	95.10	93.30

RETRACTED

**Table 4:** Bottleneck module evaluation.

Method	Training time	Precision	Recall
MSFPFN	13.5 h	93.10	90.50
MSFPFN-DR	8.9 h	93.70	92.10

## Data Availability

The datasets used during the current study are available from the corresponding author on reasonable request.
